RETRACTED

# Knockdown of lncRNA *MNX1‐AS1* suppresses cell proliferation, migration, and invasion in prostate cancer

**DOI:** 10.1002/2211-5463.12611

**Published:** 2019-04-13

**Authors:** Zongwu Li, Fangfei Wang, Shibao Zhang

**Affiliations:** ^1^ Department of Urology Jinan Central Hospital Affiliated to Shandong University China

**Keywords:** CCAT5, cell proliferation, EMT, long non‐coding RNA, *MNX1‐AS1*, prostate cancer

## Abstract

Altered expression of long non‐coding RNAs (lncRNAs) has been reported in many malignancies, including prostate cancer. However, the role of lncRNA *MNX1‐AS1* in prostate cancer has not been reported. Here, we report that *MNX1‐AS1* is expressed in prostate cancer tissues and cells and that siRNA‐mediated knockdown of *MNX1‐AS1* inhibits proliferation, migration, and invasion of prostate cancer DU145 and PC3 cells. In addition, down‐regulation of *MNX1‐AS1* decreased expression of proliferating cell nuclear antigen, PH‐3, N‐cadherin, and vimentin, but enhanced expression of E‐cadherin. In conclusion, this is the first report that knockdown of *MNX1‐AS1* suppresses prostate cancer cell proliferation, migration, and invasion. We believe that *MNX1‐AS1* may be a potential new therapeutic target for prostate cancer patients.

**Abbreviations**
CCAT5: colon cancer‐associated transcript 5
CCK‐8: Cell Counting Kit‐8
EMT: epithelial–mesenchymal transition
lncRNA: long non‐coding RNA
PCNA: proliferating cell nuclear antigen
PH‐3: phospho‐histone H3

The incidence of prostate cancer ranks second in male malignancies worldwide 1. In the USA, prostate cancer has ascended to the most common cancer in males 2. The incidence of prostate cancer in Asia is much lower than that in Europe and America, but it has been on the rise, and its growth is faster than that in developed countries 3. The risk factors for prostate cancer mainly include age, race, and heredity. New research has shown that dysfunction of steroidogenic enzyme induced by androgen stimulation, DNA methylation, and mRNA alternative splicing is crucial for the development of prostate cancer 4. Additionally, studies also found that p62, the autophagy pathway, the Hippo pathway, epigenetics, and cancer stem cells are involved in the initiation and progression of prostate cancer, and these factors may be potential targets for the treatment of prostate cancer 5. But even so, the pathogenesis of prostate cancer is still not completely known.

Long non‐coding RNA (lncRNA) is a type of non‐coding RNA molecule with a transcript length > 200 nt. LncRNA sequences are generally less conserved, but are evolutionarily conserved in promoter regions and secondary structures 6. Most of lncRNAs are generated by RNA polymerase II and have similar biological characteristics to mRNA. In physiological conditions, lncRNA interacts with microRNAs and is involved in regulating the expression of target genes 7. Numerous studies have shown that lncRNA dysfunction occurs in many malignancies, such as lung cancer 8, liver cancer 9, breast cancer 10, and colorectal cancer 11. Although lncRNA plays an important role in the proliferation, progression, metastasis, and apoptosis of tumors, the role of lncRNA in prostate cancer still remains unclear.

RETRACTED

*Lnc‐MNX1‐AS1* is located on chromosome 7, which was firstly discovered in colon cancer and so is also known as colon cancer associated transcript 5 (*CCAT5*) 12. *MNX1‐AS1* has been reported to promote cell proliferation and invasion in many malignancies 13, 14. However, the role of *MNX1‐AS1* (*CCAT5*) in prostate cancer has not been reported.

In this study, the expression level of *MNX1‐AS1* was determined in prostate cancer tissues and cells. Then, the effects of siRNA‐mediated knockdown of *MNX1‐AS1* on proliferation, migration, and invasion of prostate cancer cells were evaluated by functional experiments. To clarify the mechanism by which *MNX1‐AS1* regulates prostate cancer cell function, we further tested the expression levels of proliferating cell nuclear antigen (PCNA), phospho‐histone H3 (PH‐3), E‐cadherin, N‐cadherin and vimentin in prostate cancer DU145 and PC3 cells. We believe our study is beneficial for the diagnosis and treatment of prostate cancer.

## Materials and methods

### Patient samples

Prostate cancer samples and normal tissues were collected from patients in Jinan Central Hospital Affiliated to Shandong University. Written informed consent has been provided by each patient and the study methodologies have been approved by the Ethics Committee of Jinan Central Hospital Affiliated to Shandong University. All experiments conform to the Declaration of Helsinki.

### Cell culture and siRNA transfection

Human prostate cancer cell lines (LNCaP, DU145, PC3 and C4‐2) and a human prostate epithelial cell line (RWPE) were cultured in Dulbecco's modified Eagle's medium containing 10% FBS (Thermo Fisher Scientific, Waltham, MA, USA, 10099158) in a cell incubator at 37 °C with 5% CO_2_. siMNX1‐AS1 and scrambled siRNA plasmids were synthesized by Gene Pharma (Shanghai, China) and transfected using Lipofectamine™ RNAiMAX Transfection Reagent (Thermo Fisher Scientific, 13778030) according to the manufacturer's instructions. The transfection efficiency of the cells was detected by qRT‐PCR. Forty‐eight hours after transfection, cells were used for *in vitro* assays.

### qRT‐PCR

Total RNA was extracted with TRIzol™ LS Reagent (Thermo Fisher Scientific, 10296010) and cDNA was synthesized from RNA using the Advantage^®^ RT‐for‐PCR Kit [Takara (Dalian), Dalian, Liaoning, China, 639505]. qRT‐PCR was performed by Terra™ qPCR Direct SYBR^®^ Premix [Takara (Dalian), 638319] using a Thermal Cycler Dice™ Real Time System II [Takara (Dalian), TP900].

RETRACTED

### Detection of prostate cancer cell function

The effects of siRNA‐mediated knockdown of *MNX1‐AS1* on the cell viability of prostate cancer was performed by Cell Counting Kit (CCK‐8; Dojindo, Shanghai, China, ck‐04) according to the manufacturer's instructions and colony formation assay. The effects of siRNA‐mediated knockdown of *MNX1‐AS1* on the migration and invasion of prostate cancer cells were determined by transwell assay, with the method described by Chen *et al*. [15.

### Western blotting

Total protein was extracted from DU145 and PC3 cells using RIPA Lysis Buffer (YESEN, Shanghai, China, 20101ES60) and protein concentration was determined using the BCA Protein Assay Kit (CST, Boston, MA, USA, no. 7780). Twenty‐five micrograms of proteins was separated by 10% SDS/PAGE and then transferred to a poly(vinylidene difluoride) membrane (Millipore, Billerica, MA, USA, IPVH00010). Then, the membrane was blocked in 5% non‐fat milk for 1 h at room temperature and then incubated with the primary antibody overnight at 4 °C. The primary antibodies used were: anti‐PCNA (Abcam, ab29), anti‐histone H3 (phospho S10) (Abcam, Cambridge, UK, ab14955), anti‐E‐cadherin (Abcam, ab1416), anti‐N‐cadherin (Abcam, ab18203), anti‐vimentin (Abcam, ab8978) and anti‐glyceraldehyde 3‐phosphate dehydrogenase (GAPDH) (Abcam, ab8245). After washing three times with PBST (PBS, Tween‐20, pH7.4), the blots were incubated with secondary antibodies (Abcam, ab6721 and ab6728) at room temperature for 1 h. The poly(vinylidene difluoride) membrane was visualized by ECL assay (KeyGen, Nanjing, Jiangsu, China, KGP1128).

### Statistical analysis

All values are expressed as the mean ± SD. The two groups were compared using Student's *t*‐test. The differences between multiple groups were analyzed with one‐way analysis of variance (ANOVA) in prism 5.0 (GraphPad Software Inc., La Jolla, CA, USA). *P *<* *0.05 was considered statistically significant.

## Results

### *MNX1‐AS1* is up‐regulated in prostate cancer tissues and cell lines

We determined the expression level of *MNX1‐AS1* in prostate cancer tissues and adjacent normal tissues (*n* = 70) using qRT‐PCR. As shown in Fig. 1A, the expression of *MNX1‐AS1* mRNA was significantly up‐regulated in tumor tissues compared with corresponding normal tissues (*P *<* *0.001). Next, several human prostate cancer cell lines (LNCaP, DU145, PC3 and C4‐2) and one human prostate epithelial cell line (RWPE) were used to detect the expression of *MNX1‐AS1* mRNA. The results showed that the expression level of *MNX1‐AS1* in tumor cells (LNCaP, DU145, PC3, and C4‐2) was significantly higher than that in RWPE cells (*P *<* *0.01; Fig. 1B). These results indicate that *MNX1‐AS1* may be a prognostic and therapeutic biomarker in prostate cancer patients.

RETRACTED

**Figure 1:** *MNX1‐AS1* is up‐regulated in prostate cancer. (A) The expression of *MNX1‐AS1* was determined by qRT‐PCR in prostate tumor tissues and adjacent normal tissues (*n* = 70). Data were plotted using prism 5.0. ***P <* *0.001, compared with adjacent tissues, Student's *t*‐test. (B) The expression of *MNX1‐AS1* was determined by qRT‐PCR in human prostate cancer LNCaP, DU145, PC3 and C4‐2 cell lines and human prostate epithelial RWPE cell. Data were processed with prism 5.0. All values are expressed as mean ± SD. **P <* *0.01, ***P <* *0.001, compared with RWPE cells, one‐way ANOVA.

### Down‐regulation of *MNX1‐AS1* inhibits prostate cancer cell proliferation

To further explore the effects of *MNX1‐AS1* on prostatic cancer cell function, two specific siRNAs (siMNX1‐AS1#1 and siMNX1‐AS1#2) were used to knock down *MNX1‐AS1*, and their efficiency was tested in prostatic cancer DU145 and PC3 cells (Fig. 2A). Then, the cell viability of DU145 and PC3 cells transfected with *MNX1‐AS1* siRNAs or negative control siRNA was evaluated using the CCK‐8 assay. As shown in Fig. 2B, the prostatic cell viability was significantly inhibited by down‐regulation of *MNX1‐AS1* compared with the control group (*P *<* *0.001). Then, we performed a colony formation assay, and the results showed that knocking down *MNX1‐AS1* effectively inhibited the formation of colonies derived from DU145 and PC3 prostatic cells compared with the control group (*P *<* *0.001; Fig. 2C). Thus, these data revealed that *MNX1‐AS1* is able to promote cell proliferation in prostate cancer.

**Figure 2:** Down‐regulation of *MNX1‐AS1* inhibits the proliferation of prostate cancer cells. (A) The silencing efficacy of *MNX1‐AS1* was measured by qRT‐PCR in DU145 and PC3 cells. Data were processed with prism 5.0. All values are expressed as mean ± SD. **P <* *0.01, ***P <* *0.001, compared with siNC, one‐way ANOVA. (B) CCK‐8 assay was used to detect the viability of DU145 and PC3 cells transfected with siR‐MNX1‐AS1. Data were plotted with prism 5.0. All values are expressed as mean ± SD. ***P <* *0.001, compared with siNC, one‐way ANOVA. (C) Clone formation assay was used to detect the viability of DU145 and PC3 cells transfected with siR‐MNX1‐AS1. Data were processed with prism 5.0. All values are expressed as mean ± SD. ***P <* *0.001, compared with siNC, Student's *t*‐test.

RETRACTED

### Down‐regulation of *MNX1‐AS1* inhibits prostate cancer cell migration and invasion

The migration and invasion of prostatic cells seriously affect the prognosis and survival of prostate patients. Next, a transwell assay was performed to determine whether *MNX1‐AS1* affected the migratory and invasive potential of prostatic cancer cells. Firstly, the number of prostatic cells passed through the transwell membrane was observed to be reduced by siRNA‐mediated knockdown of *MNX1‐AS1*, suggesting that down‐regulation of *MNX1‐AS1* could inhibit prostatic cancer cell migration *in vitro* (*P *<* *0.01; Fig. 3A). Moreover, the transwell invasion assay also showed that suppression of *MNX1‐AS1* could significantly restrain the invasive ability of DU145 and PC3 cells (*P *<* *0.01; Fig. 3B).

**Figure 3:** Down‐regulation of *MNX1‐AS1* inhibits the migration and invasion of prostate cancer cells. (A) Transwell assay was performed to analyze the migration of DU145 and PC3 cells transfected with siR‐MNX1‐AS1. Data were processed with prism 5.0. Scale bar = 2.5 μm. All values are expressed as mean ± SD. **P <* *0.01, compared with siNC, one‐way ANOVA. (B) Transwell assay was performed to analyze the invasion of DU145 and PC3 cells transfected with siR‐MNX1‐AS1. Data were processed with prism 5.0. Scale bar = 2.5 μm. All values are expressed as mean ± SD. **P <* *0.01, compared with siNC, one‐way ANOVA.

### *MNX1‐AS1* regulates the expression of related mRNAs and proteins in prostate cancer cells

Having proven that knockdown of *MNX1‐AS1* was able to inhibit the proliferative, migratory, and invasive ability of prostate cancer cells, we then explored the specific mechanism. At first, the mRNA expression level of PCNA and PH‐3 was tested after knocking down *MNX1‐AS1* in DU145 and PC3 cells. The results indicated that these proliferative markers were observably decreased by knockdown of *MNX1‐AS1* at the mRNA level compared with NC cells, which suggested that *MNX1‐AS1* might promote the proliferation of prostate cancer cells via regulating PCNA and PH‐3 (Fig. 4A). Epithelial–mesenchymal transition (EMT) is critical for cell migration and invasion of prostate cancer, and E‐cadherin, N‐cadherin and vimentin are the markers of EMT. We also found knockdown of *MNX1‐AS1* promoted E‐cadherin mRNA expression whereas it inhibited N‐cadherin and vimentin mRNA expression in DU145 and PC3 cells compared with the control, indicating that *MNX1‐AS1* might induce the migration and invasion of prostate cancer cells via regulating EMT (Fig. 4A). Similarly, results from western blotting also showed that the protein expression of PCNA, PH‐3, N‐cadherin and vimentin was reduced significantly, but the E‐cadherin expression was enhanced by down‐regulation of *MNX1‐AS1* in DU145 and PC3 cells (Fig. 4B).

RETRACTED

**Figure 4:** *MNX1‐AS1* regulates the expression of related mRNAs and proteins in prostate cancer cells. (A) The mRNA expressions of PCNA, PH‐3, E‐cadherin, N‐cadherin and vimentin in DU145 and PC3 cells transfected with siR‐MNX1‐AS1. Data were processed with prism 5.0. All values are expressed as mean ± SD. *P <* *0.05, **P <* *0.01, ***P <* *0.001, compared with siNC, one‐way ANOVA. (B) The protein expressions of PCNA, PH‐3, E‐cadherin, N‐cadherin and vimentin in DU145 and PC3 cells transfected with siR‐MNX1‐AS1. Data were processed with prism 5.0.

## Discussion and conclusion

Although it is known that lncRNA plays a crucial role in gene regulatory processes and it is closely related to the pathogenesis of various cancers 16, the relationship between lncRNA and prostate cancer is still poorly understood. *CCAT* is a type of lncRNA first discovered in colon cancer, named *CCAT1*,* CCAT2*,* CCAT3*,* CCAT4*, and *CCAT5* (namely *MNX1‐AS1*) according to the order of discovery. Dysregulation of *CCAT* has been shown in various types of cancers 17. Jiang *et al*. 18 reported that activation of *CCAT1* by TP63 and SOX2 was able to promote squamous cancer progression. Li *et al*. 19 found that silencing of *CCAT1* inhibits cell proliferation, invasion, and peritoneal metastasis via down‐regulating *Bmi‐1* in gastric cancer. Notably, Liu *et al*. 20 reported that *CCAT1* can restrain prostate cancer migration via altering macrophage polarization. However, the biological functions and mechanisms of *CCAT5*/*MNX1‐AS1* in prostate cancer have not been reported.

In the present study, we compared the differences in expression level of MNX1‐AS1 between prostate cancer and normal prostate tissues/cells and found that MNX1‐AS1 was significantly up‐regulated in prostate cancer (Fig. 1). Related studies demonstrated that lncRNA plays a key role in cell proliferation of prostate cancer 21. We performed a CCK‐8 assay (Fig. 2B) and clone formation assay (Fig. 2C) to detect prostate cancer cell proliferation after knocking down MNX1‐AS1, and found that MNX1‐AS1 plays a significant role in proliferation of prostate cancer DU145 and PC3 cells, which was in agreement with the previous research 21. Additionally, it was reported that up‐regulation of *CCAT1* could promote EMT in several malignancies, including prostate cancer 22. As well, results from the transwell assay showed that MNX1‐AS1 is crucial for prostate cancer cell migration (Fig. 3A) and invasion (Fig. 3B).

RETRACTED

We wanted to know how MNX1‐AS1 regulates prostatic cancer cell function. PCNA is synthesized in the nucleus and is an accessory protein of DNA polymerase δ 23. PCNA is closely related to cellular DNA synthesis and is a good biomarker for cell proliferation 24. PH‐3 has a temporal and spatial correlation with chromosome agglutination and deagglutination during cell mitosis 25. In this study, the expression of PCNA and PH‐3 was observably decreased after knocking down *MNX1‐AS1* at both the mRNA and the protein level, indicating that *MNX1‐AS1* might promote the proliferation of prostate cancer cells via targeting PCNA and PH‐3. In addition, Søgaard *et al*. 26 reported that targeting PCNA has the potential to improve docetaxel therapy for prostate cancer, suggesting that down‐regulation of *MNX1‐AS1* might be a potential therapeutic strategy for prostatic cancer.

Prostate cancer‐related deaths are often caused by metastasis of tumor cells, and EMT plays an important role in tumor metastasis 27. The main features of EMT include the abnormal expressions of cell adhesion molecules (E‐cadherin and N‐cadherin) and the transformation of cytokeratin into vimentin 28, 29. Through EMT, epithelial cells lose the attachment to the basement membrane and obtain more interstitial phenotypes such as high migration and invasion, anti‐apoptosis, and the ability to degrade the extracellular matrix 30. This study also showed that knockdown of *MNX1‐AS1* promoted E‐cadherin expression whereas it inhibited expression of N‐cadherin and vimentin in prostate cancer cells, indicating that *MNX1‐AS1* might promote the migration and invasion of prostate cancer cells via regulating EMT. In summary, this is the first report showing that knockdown of *MNX1‐AS1* restrains prostate cancer cell proliferation, migration, and invasion. We believe our finding has positive clinical significance in prostate cancer therapy.

## Conflict of interest

The authors declare no conflict of interest.

## Author contributions

ZL and FW conducted experiments and were responsible for data acquisition, analysis, interpretation, and manuscript writing. SZ conceived and designed the study, and revised the manuscript critically for important intellectual content. All authors read and approved the final manuscript.
